# Assessment of immediate and non-immediate hypersensitivity contrast reactions by skin tests and provocation tests: A review

**DOI:** 10.1177/20587384211015061

**Published:** 2021-05-31

**Authors:** Rakesh D Bansie, A Faiz Karim, Maurits S van Maaren, Maud AW Hermans, Paul LA van Daele, Roy Gerth van Wijk, Saskia M Rombach

**Affiliations:** 1 Department of Internal Medicine, Section Allergy and Clinical Immunology, Erasmus Medical Center, Rotterdam, Zuid-Holland, the Netherlands; 2 Department of Internal Medicine, Academic Hospital Paramaribo, Paramaribo, Suriname; 3 Department of Internal Medicine, Section Allergy and Clinical Immunology, Gouda Groene Hart Ziekenhuis, Zuid-Holland, the Netherlands

**Keywords:** allergy, contrast, gadolinium contrast media, hypersensitivity reaction, immediate hypersensitivity reaction, iodinated contrast media, non-immediate hypersensitivity reaction, provocation, skin test

## Abstract

**Introduction:**

Allergic and nonallergic hypersensitivity reactions to iodinated contrast media (ICM) and gadolinium-based contrast media are classified as immediate or non-immediate hypersensitivity reactions (IHR and NIHR), respectively. Skin tests and provocation tests are recommended for the evaluation of hypersensitivity reactions to contrast agents; however provocations are not common in clinical practice.

**Methods:**

A MEDLINE search was conducted to investigate studies comprising both skin tests and provocation tests that evaluated hypersensitivity reactions to ICM.

**Results:**

Nineteen studies were identified that reported on skin tests, followed by provocations. In the case of IHR to ICM, 65/69 (94%) patients with a positive skin test for the culprit media tolerated a challenge with a skin-test-negative alternative ICM. In IHR to ICM with a negative skin test for the culprit media, provocations were positive in 3.2%–9.1% patients. In the case of a NIHR to ICM with a positive skin test, provocation with a skin-test-negative agent was tolerated in 75/105 (71%) of cases. In NIHR with a negative skin test for the culprit agent, re-exposure to the culprit or an alternative was positive in 0%–34.6% patients. Provocations with the same ICM in skin test positive patients with IHR or NIHR were positive for a majority of the patients, although such provocation tests were rarely performed. Data on hypersensitivity reactions, skin tests and provocations with gadolinium-based contrast media were limited; however, they exhibited a pattern similar to that observed in ICM.

**Conclusion:**

In both ICM and gadolinium-based contrast media, the risk of an immediate repeat reaction is low when skin tests are negative. In contrast, a provocation with a skin-test-positive contrast medium showed a high risk of an immediate repeat hypersensitivity reaction. Therefore, a thorough medical history is necessary, followed by skin tests. A provocation is recommended, for diagnostic work-up, when the diagnosis is uncertain.

## Introduction

Iodinated contrast media (ICM) and gadolinium-based contrast media are essential for radiographic imaging in current medical practice. ICM is annually used in over 75 million procedures worldwide.^1^ Following the introduction of the MRI, gadolinium-based MR agents have been used.^2^

Hypersensitivity reactions may occur in patients upon administration of the contrast media. The first large prospective survey in 1975 on ICM-induced hypersensitivity reactions showed an overall incidence of contrast reactions in 2.33%–5.65% patients.^3^ Recent numbers vary from 1% to 12% and severe reactions, mainly anaphylaxis, comprise 0.01% to 0.2% of all reactions.^4–6^ Hypersensitivity reactions were more frequently observed with high osmolar contrast agents than with low osmolar contrast agents, that is approximately 15% versus 3% respectively. This has led to the reduced use of high osmolar agents over the years.^7^ Iodixanol (Visipaque^®^) and iohexol (Omnipaque^®^) are both low osmolar ICMs and are commonly used in clinical practice nowadays.

Moreover, severe reactions are also less common with the use of nonionic ICM than with ionic ICM.^8^

Further, hypersensitivity reactions against gadolinium are less common, with an estimated prevalence of 0.07%–2.4%.^9^

Reactions observed during or after administration of ICM and gadolinium-based contrast media are clinically divided into three categories: hypersensitivity reactions, pharmacological toxicity and events unrelated to contrast media exposure, including other allergens other than the contrast media.^2,8^ The term hypersensitivity is used to describe objectively reproducible symptoms or signs initiated by exposure to a defined stimulus (i.e. contrast agent), at a dose normally tolerated in people.^10^ Hypersensitivity reactions can be an allergic hypersensitivity or a non-allergic hypersensitivity reaction.^10^ Furthermore, hypersensitivity reactions are classified as either immediate (IHR) or non-immediate reactions (NIHR).^8^ Immediate reactions to ICM or gadolinium-based contrast media occur within 1 h; however they have been reported to occur up to 6 h after exposure and are based on either IgE-mediated or non-IgE-mediated hypersensitivity.^11^ The latter is thought to occur due to direct activation of basophilic granulocytes and mast cells because of the hyperosomolar nature of older types of radiocontrast media, or via complement anaphylatoxins C3a and C5a.^12^ Although most IHRs are non-allergic, in case of a severe IHR to ICM the patient is more likely to have an IgE-mediated reaction.^8^ It is important to note that hypersensitivity reactions in ICM are not due to hypersensitivity to iodine but to the chemical structure of ICM. For instance, there is no cross-reactivity between ICM hypersensitivity reactions and shellfish or povidone-iodine allergies.^13,14^ Lastly, in contrast to popular belief, clonal mast cell disorders are not a risk factor for radiocontrast media hypersensitivity, as previously stated in the AAAAI Work Group Report last year.^15^

Non-immediate hypersensitivity allergic reactions are T cell-mediated type IV hypersensitivity reactions.^8,16^ NIHR can develop after 1 h or even after 7 days and can persist for 1–7 days.^8^ The frequency of NIHR ranges from 0.5% to 23% for ICM.^17^ The NIHRs to gadolinium are probably not common as there are only a few published cases. These reactions usually present with maculopapular exanthema.^8^ Although rare, NIHR such as DRESS, Stevens-Johnson syndrome and toxic epidermal necrolysis have been reported.^8^

To evaluate whether there is an allergic hypersensitivity reaction, skin prick tests (SPT) and intradermal tests (IDT) including non-immediate reading (after 48 h) should be performed, between 1 and 6 months after the hypersensitivity reaction.^18–22^ Drug provocation tests are recommended in addition to skin tests for hypersensitivity reactions to radiocontrast agents.^23^ However, radiocontrast agent provocations are recommended based on a risk benefit analysis^11^ and are suggested to confirm the tolerability of radiocontrast media after a very severe reaction in case of a negative skin test.^24^ Provocations are not common in clinical practice and practical guidelines are lacking.

The aim of this literature review is to evaluate the added value of a provocation test, in addition to skin tests, for the assessment of immediate and non-immediate hypersensitivity contrast reactions. We performed extensive literature review and data analysis and prepared a flow chart, to optimize the diagnostic evaluation of hypersensitivity reactions to iodine and gadolinium-based contrast media, including provocation tests.

## Methods

### Review of the literature

A literature search was conducted using MEDLINE, which was finalised on 21st of December 2020. The title and abstract [tiab] were screened to identify studies addressing the value of the provocation test in addition to skin tests. The search terms used were as follows: (hypersensitivity [tiab] AND contrast [tiab] AND test [tiab]) OR (hypersensitivity [tiab] AND radiocontrast [tiab] AND test [tiab]). Further, the search was repeated using allergy instead of hypersensitivity.

#### Inclusion criteria

We included studies that described any type of skin tests as well as a provocation test or follow-up with a re-exposure to contrast media in the evaluation of an immediate hypersensitivity reaction (IHR) and/or a non-immediate hypersensitivity reaction (NIHR) for patients with a history of hypersensitivity reactions to contrast media.

#### Exclusion criteria

Research articles and reviews published in languages other than English were excluded. Studies reporting only skin tests without re-exposure to contrast media or a provocation test were excluded.

The titles and abstracts of the articles were screened by two independent reviewers (RB and SR) who applied the inclusion and exclusion criteria. Consensus was reached; therefore the opinion of a third reviewer was not required.

### Analysis

Data from the included studies were assessed based on the results of the provocation tests or re-exposure of contrast media in relation to the skin tests (SPT, IDT, patch test) for contrast hypersensitivity. Provocation or re-exposure consisted of the (re-)introduction of the culprit or alternative radio-contrast agent in patients with a negative skin test, the introduction of a skin test negative radio-contrast agent in patients with positive skin tests or the reintroduction of a skin-test positive radio-contrast agent in patients with a positive skin test.

Hypersensitivity reactions were categorised as IHR and NIHR. The studies that included both IHR and NIHR were re-assessed and extracted as data for IHR and NIHR. The distinction between IHR and NIHR was based on the corresponding clinical presentation and results from the performed skin tests (SPT, IDT or patch test). Patch tests are generally performed to analyse non-immediate hypersensitivity reactions. Delayed readings were also reported for SPT and IDT which were then correlated with the clinical presentation.^18,25,26^

Studies were assessed based on the outcome of provocation or re-exposure to a radio-contrast agent.

The negative predictive value was calculated as follows:

the number of negative skin tests followed by a negative provocation/(number of negative skin tests followed by positive and negative provocations).

The positive predictive value was calculated as follows:

the number of positive skin tests followed by a positive provocation/(number of positive skin tests followed by positive and negative provocations).

## Results

The literature search identified 508 studies, of which 19 studies were included, after screening the title and abstract, and applying the inclusion criteria (Figure 1). One study was excluded from the analysis as patients without previous contrast hypersensitivity reactions or previous exposure to contrast media were included.^27^ Another study was excluded, as the results of the provocation data were combined for patients with a previous history of hypersensitivity reactions and controls without a previous contrast reaction.^28^

**Figure 1.** Flow-chart of study selection after application of search terms.

Fourteen studies reported on the outcomes of iodinated contrast-based reactions, four on gadolinium-based reactions and one published on both. Eleven out the 19 studies were retrospective studies. The results are shown in Tables 1 to 4.

**Table 1.** Patient characteristics of included studies with ICM (*n* = 14 studies). Severity of symptoms was reported as mild, moderate or severe or grade I, II, III, IV, corresponding to increasing severity.

Author	*N*	F/M	Age (median, range) or mean ± SD	IHR	NIHR	Unknown type of reaction	Symptoms/severity IHR: events	Symptoms/severity NIHR: (number of reactions)
Vernassiere et al.^53^	15	11/4	55.4 (37–78)	NA	15	–	NA	MPE: 5
								Macular rash: 5
								Pruritus: 1
								Pompholyx: 1
								Erythema/edema: 3
Seitz et al.^25^	32	17/15	48 (24–71)	NA	32	–	NA	Exanthema gr.I: 7
								Exanthema gr. II: 20
								Exanthema gr. III: 5
Caimmi et al.^54^	120	75/45	56 (45–65)	101/120	17	2	Gr. I: 42	Mild: 1
							Gr. II: 34	Moderate: 16
							Gr. III: 20	
							Gr. IV: 5	
Torres et al.^29^	161	79/82	58.5 (IQR 48.85–66.5)	NA	161	–	NA	Mild: 16
								Moderate:143
								Severe: 2
Salas et al.^30^	90	63/27	54.50 ± 27	90	*NA*	–	Gr. I: 69	NA
							Gr. II: 18	
							Gr. III: 3	
Prieto-Garcia et al.^55^	106	64/42	56.7 ± 16.9	106	*NA*	–	Gr. I: 66	NA
							Gr. II: 29	
							Gr. III: 11	
Ahn et al.^21^	23	13/10	48.6 ± 14.8	17	6	–	Anaphylaxis: 10	MPE: 23
							Urticarial: 7	
Della-Torre et al.^31^	36	27/9	58 (22–75)	19	17	–	Gr. I: 12	Mild 16
							Gr. II: 3	Moderate: 1
							Gr. III: 4	
Sese et al.^56^	37	24/13	49.3	37	NA	–	Gr. I: 26	NA
							Gr. II: 4	
							Gr. III: 7	
Schrijvers et al.^18^	597	406/191	60 (13–92)	423	118	56	Gr. I: 122	Not severe: 109
							Gr. II: 104	Severe: 9
							Gr. III + IV: 100	
Trautmann et al.^26^	45	30/15	55-58 (20–80)	11/32	13	–	Mild: 20	MPE: 11
							Mod: 7	Systemic: 1
							Severe: 5,	FDE: 1
Kwon et al.^32^	69	40/29	58.8 ± 10.9	69	NA	–	Mild: 25	NA
							Mod: 5	
							Severe: 39	
Meucci et al.^33^	98	53/45	65.6 (23–90)	82	16	–	Gr. I: 47	Mild: 15
							Gr. II:24	Moderate: 1
							Gr. III: 10	
							Gr. IV: 0	
Dona et al.^34^	101	52/49	62 (IQR 49–69)	12	89	–	Gr. I: 7	Maculopapular exanthema: 60
							Gr. II: 2	
							Gr.III:3	Delayed urticaria:29
							Gr. IV:0	

NA: not applicable; F: female; M: male; Gr: grade; MPE: maculopapular exanthema; FDE: fixed drug eruption; IQR: interquartile range.

**Table 2.** Provocation/re-exposure of ICM in patients with an immediate hypersensitivity reaction (IHR) (*n* = 11 studies).

Author	Study design	*N* (IHR)	Direct positive SPT or IDT (%)	Culprit skin test negative		Culprit skin test positive				Premedication administered prior to provocation or re-exposure
				Positive provocation test or re-exposure reaction to culprit or skin test negative alternative ICM (%)	Negative predictive value	Positive provocation test or exposure reaction to skin test negative ICM (%)	Negative predictive value	Positive provocation test or exposure reaction to skin test positive ICM (%)	Positive predictive value	
Caimmi et al.^54^	R	101	17/101 (16.8)	1/23 (4.4)	0.96	0/1 (0)	1	–	NA	None
Salas et al.^33^	P, I	90	5/90 (5.6)	3/74 (4.1)	0.96	2/4 (50)^a^	0.5	–	NA	None
Prieto-Garcia et al.^55^	P, I	106	11/106 (10.4)	–	NA	0/7 (0)	1	–	NA	None
Ahn et al.^21^	P	17	11/17 (64.7)	–	NA	0/2 (0)	1	2/2 (100)	1	In all
Della-Torre et al.^31^	R	19	7/19 (36.8)	1/12 (8.3)	0.92	0/7 (0)	1	–	NA	In all
Sesé et al.^56^	R,I	37	5/37 (13.5)	1/31 (3.2)	0.97	0/5 (0)	1	–	NA	None
Schrijvers et al.^18^	R	423	56/423 (13.2)	8/159 (5.3)^b^	0.95	0/9^c^ (0)	1	–	NA	In 31/150
Trautmann et al.^26^	R	32	11/32 (34.4)	–	NA	0/10 (0)	1	–	NA	None
Kwon et al.^32^	R	69	38/69 (55.0 )	2/22 (9.1)	0.91	0/11 (0)	1	4/5 (80)	0.8	None
Meucci et al.^33^	R	82	7/82 (8.5)	3/75 (4)	0.96	0/7 (0)	1	–	NA	None
Dona et al.^34^	P	12	6/12 (50)	6/6 (100)^d^	0	2/6 (33)	0.67	–	NA	None

N: number of patients; P: prospective; R: retrospective; I: intervention; NA: not applicable.

a One case was excluded in which iobitridol was provocated, but a basophil activation test was performed instead of a skin test.

b Two cases in the group of patients with IHR and with negative skin tests and a positive reaction upon provocation were excluded due to the provocation with an unknown ICM.

c Two cases in the group of patients with IHR and positive skin tests and with a positive reaction upon provocation were excluded due to the provocation with an unknown ICM.

d Patients with a proven ICM allergy, based on clinical history, skin tests and drug provocation tests, were evaluated for an allergy to another ICM.

**Table 3.** Provocation/re-exposure of ICM in patients with a non-immediate hypersensitivity reaction (NIHR) (*n* = 10 studies).

Study	Study design	*N* (NIHR)	(Delayed) Positive SPT and/or IDT or patch test (%)	Culprit skin test negative		Culprit skin test positive				Premedication administered prior to provocation or re-exposure
				Positive provocation test or re-exposure reaction to culprit or skin test negative alternative ICM (%)	Negative predictive value	Positive provocation test or exposure reaction to skin test negative ICM (%)	Negative predictive value	Positive provocation test or exposure reaction to skin test positive ICM (%)	Positive predictive value	
Vernassiere et al.^53^	R, I	15	8/15 (53.3)	2/7 (28.6)	0.71	3/8 (37.5)	0.625	–	NA	None
Seitz et al.^25^	R, I	32	6/32 (18.8)	–	NA	0/4 (0)	1	–	NA	None
Caimmi et al.^54^	R	17	3/17 (42.9)	1/4 (25)	0.75	–	NA	–	NA	None
Torres et al.^29^	P, I	161	34/161 (21.1)	44/127 (34.6)	0.65	11/34 (32.4)	0.68	–	NA	None
Ahn et al.^21^	P	6	3/6 (50)	–	NA	0/1 (0)	1	–	NA	In all
Della-Torre et al.^31^	R	17	5/17 (29.4)	0/12 (0)	1	0/5 (0)	1	–	NA	In all
Schrijvers et al.^18^	R	118	20/118 (16.9)	5/37(12.8)^a^	0.86	0/4^a^ (0)	1	1/2^a^ (50)	0.5	In 20.7%
Trautmann et al.^26^	R	13	13/13 (100)	–	NA	0/8 (0)	1	–	NA	None
Meucci et al.^33^	R	16	3/16 (18.8 )	4/13 (30.8)	0.69	2/2 (100)	0	1/1 (100)	1	None
Dona et al.^34^	P	89	39/89 (43.8)	50/50 (100)^b^	0	14/39 (35.9)	0.64	–	NA	None

N: number of patients; P: prospective; R: retrospective; NA: not applicable.

a Five patients had a positive skin test. One with NIHR and positive skin tests and with a positive reaction upon provocation was excluded due to the provocation with an unknown ICM.

b Patients with a proven ICM allergy, based on clinical history, skin tests and drug provocation tests, were evaluated for an allergy to other ICM.

**Table 4.** Provocation/re-exposure to gadolinium contrast media (*n* = 4 studies).

Study	Study design	*N*	Immediate reactions	Non-immediate reaction	Culprit skin test negative		Culprit skin test positive				Premedication administered prior to provocation or re-exposure (%)
			Positive SPT or IDT (%)	Positive patch test/SPT and/or IDT (%)	Positive provocation test with culprit or skin test negative alternative GCM (%)	Negative predictive value	Positive provocation with skin test negative GCM (%)	Negative predictive value	Positive provocation with skin test positive GCM	Positive predictive value	
Chiriac et al.^35^	P	27	5/26 (19.2)	0/1 (0)	0/10 (0)	1	0/1 (0)	1	–	NA	3/6 (50)
Moulin et al.^36^	P	1	1/1	–	–	NA	0/1 (0)	1	–	NA	NR
Kolenda et al.^37^	R	33	19/33 (57.6)	–	0/9 (0)	1	0/11 (0)	1	–	NA	NR
Seta et al.^38^	R, I	14	3/12 (25)	0/1 (0)	2/11 (18.2)	0.82	0/1 (0)	1	–	NA	NR

N: number of patients; P: prospective; R: retrospective; I: intervention; NA: not applicable; NR: not reported.

Repeating the search using the term ‘allergy’ instead of ‘hypersensitivity’ did not reveal any other study that fulfilled the inclusion criteria.

### Iodinated contrast media

Seven studies included skin tests and provocation/re-exposure to ICM for both IHR and NIHR to ICM, four studies assessed IHR for ICM and three studies assessed NIHR for ICM (Table 1).

Standard pre-medication before provocation was administered in two studies.^21,31^ In another study pre-medication was used in a subgroup consisting of patients, including those with mast cell disorders or chronic urticaria who had negative skin tests,^18^ Table 2.

Most studies included more women than men. The median and mean age of the patients was between 48 and 62 years. Severe reactions for IHR and NIHR were not reported frequently (Table 1). Most studies used the Ring and Messmer grading scale for IHR: grade 1, generalised (muco)cutaneous symptoms; grade 2, mild systemic manifestations; grade 3, life-threating systemic reactions including shock and grade 4, cardiac or respiratory arrest (Table 1).

#### Immediate hypersensitivity reactions to ICM

Skin prick tests or intradermal tests were positive in 5.6%–64.7% patients with IHR (Table 2). In the case of a negative skin test, provocation with the culprit or a negatively tested alternative was positive in 3.2%–9.1% patients (Table 2). However, in one study with six skin-test-negative patients and confirmed immediate hypersensitivity to another ICM all provocation tests were positive for the alternative.^34^ More-over in the 11 studies performed, 65 of 69 (94%) patients with a positive skin test with the culprit ICM tolerated a challenge with a skin-test-negative alternative ICM. Two out of four patients in one study^30^ as well as two out of six patients in another study,^34^ with positive skin tests for the culprit media and challenged with a negative-skin-test alternative ICM, experienced symptoms during provocation, Table 2. Dona et al.^34^ reported that the symptoms were similar to those recorded earlier, however they were milder .

Provocations with the culprit ICM are rarely performed in cases with a positive skin test. Only two studies addressed this issue and positive provocation tests were seen in 4/5 and 2/2 patients respectively.^21,32^

#### Non-immediate hypersensitivity reactions to ICM

Skin prick tests, intradermal tests or patch tests were positive in 16.9%–53.3% of patients with NIHR (Table 3). In case of a negative skin test for the culprit or alternative ICM, provocation with the tested ICM was positive in 0%–34.6% of cases and in 50/50 (100%) patients challenged with the skin-test negative culprit with a proven non-immediate type allergic sensitivity to another ICM (Table 3). In case of a NIHR with a positive skin test, provocation with an alternative skin test negative agent was tolerated in 75/105 (71%) of cases Table 3. Provocation with the culprit was rarely performed when the skin test was positive, resulting in a hypersensitivity response in two out of three patients.^18,33^

### Gadolinium based contrast media

In gadolinium-based contrast media, one case report and three case series reported a positive skin test in 19.2%–57.6% of patients that had an IHR (Table 4). Limited information was available for NIHR.

In the case of IHR with positive skin tests, a provocation was performed with an alternative gadolinium-based contrast medium and a negative skin test: all provocations were negative.^35–38^

In the case of a negative skin test, provocations with the culprit or alternative ICM were negative in all the studies with the exception of one study that reported two positive provocation results in 11 cases, one with an immediate and one with a non-immediate hypersensitivity reaction (Table 4). However, the severity of the response was not mentioned.^38^

One study reported on patients that had hypersensitivity reactions to ICM or gadolinium-based contrast media.^39^ Of the 10 patients with an IHR and three with a NIHR, none showed a positive skin test. Of those, one patient with a previous NIHR response to ICM, tolerated the gadolinium-based contrast medium.

## Discussion

Radiocontrast media provocation tests are recommended in addition to skin tests, although these are not common in clinical practice. A recent study suggests a provocation based on a risk benefit analysis.^11^ In another recently published algorithm on contrast reactions, a negative skin test radiocontrast provocation is only recommended as a confirmation test for tolerability in case of very severe reactions.^24^ However, a radiocontrast provocation could also be useful to differentiate an allergic hypersensitivity reaction from non-allergic hypersensitivity reactions and in case of less severe reactions.

In the studies in this review, provocations were mostly performed when a computerized tomography (CT) scan or MRI was needed and re-exposure to the contrast agent was indicated. The results of this review indicated that when the skin test was positive, provocation testing with the same agent as the culprit agent was positive in most cases, also reflected by the high positive predictive value of the skin test. Because these DPTs were positive in most cases, positive skin tests may represent/indicate a true allergy. A skin test can be positive in patients without previous exposure to contrast media, even if provocation with this particular contrast medium afterwards is well tolerated.^27^ This illustrates that the clinical symptoms should be compatible with a hypersensitivity reaction for accurate interpretation of the skin test results, and a provocation can be of additional value in cases where the history of the patient and results of the skin test do not match.

In case of IHR and NIHR to ICM, the majority of patients (94% and 71% respectively) with a positive skin test for the culprit tolerated a challenge with a skin-test-negative alternative ICM. In case of a negative skin test for the culprit, provocations were mostly negative, as reflected by the high negative predictive value of the skin test, although the number of positive provocations was higher in the NIHR group. This variation can be explained by the number of patients in the studies, the inclusion of patients with varying numbers of allergic and non-allergic hypersensitivities and time and type of skin test performed. The risk of a NIHR, despite a provocation with a negative skin test ICM, is probably more around the 34.6% as reported in the study with the highest number of patients.^29^

A previous reaction to ICM is the most common risk factor for IHR.^4,8,40,41^ Although cross-reactivity is relatively low for ICM in immediate hypersensitivity reactions,^1^ the risk of a hypersensitivity reaction is higher in patients with a confirmed allergic ICM hypersensitivity, even with a negative skin test.^34^

Higher degrees of cross reactivity, ranging from 32% to 75%, with skin tests for ICM were seen with NIHR.^22,42^ Therefore it is recommended to perform an additional provocation, in case of a proven allergy, even when the skin test for the alternative contrast agent is negative.

Other risk factors for IHR are asthma, use of beta-blockers, old age and cardiovascular diseases.^4,8,41,43–46^ Reported predisposing factors for NIHR are previous CM-induced hypersensitivity reactions, atopy, interleukin-2 treatment, serum creatinine level >2 mg/dL and a history of drug and contact allergy.^8,47,48^

Data on hypersensitivity reactions, skin tests and provocation tests for gadolinium-based contrast media were scarce; however they showed a similar pattern to the hypersensitivity reactions in ICM. There is no cross-reactivity between ICM and gadolinium contrast media.^49^

When an allergic hypersensitivity reaction, evaluated by skin tests and a provocation, is excluded, it is generally considered as a non-allergic hypersensitivity reaction, or a reaction not related to the contrast media itself. Apart from hypersensitivity reactions, common side effects occurring immediately after administration of ICM include flushing, vomiting and occasionally dyspnea. Assessing the concentration of tryptase between 0.5 and 3 h after the onset of symptoms may help to determine the cause of the reaction.^50^ An elevated tryptase level is indicative of a mast cell-mediated reaction and increases the probability of an IgE-mediated allergic reaction.^51^ Although a high tryptase is associated with more severe immediate hypersensitivity reactions, a normal tryptase level does not exclude an IHR.^50^ After 1–2 days, a plasma tryptase level can be drawn for baseline analysis.^52^

Based on this review and other studies from the literature on this topic, the following diagnostic approach for the evaluation of a hypersensitivity reaction to contrast media is proposed:

In case of an immediate hypersensitivity reaction, the serum tryptase level should be measured between 15 and 180 min after the reaction. An increase in tryptase, particularly when confirmed with a positive skin test is suggestive of an IgE-mediated hypersensitivity reaction. A repeat measurement of tryptase at least 1 or 2 days later is useful to confirm normal baseline values. Otherwise, a thorough medical history is necessary, followed by an undiluted skin prick test and if negative subsequently an intradermal test with a dilution of 1:10 in case of iodine contrast media. In additional, an undiluted IDT can be performed in case of a non-immediate type hypersensitivity reaction for optimal sensitivity.^18,29,34^

For gadolinium-based hypersensitivity reactions, IDT including dilutions of 1:1000, 1:100 and 1:10 are recommended.^35,37^

Patients with a positive skin test and the history of hypersensitivity reaction are classified as allergic (Figure 2).

**Figure 2.** Proposed flow-chart for assessment of presumed contrast hypersensitivity.

However, when the skin test is negative, a provocation with the alternative media should be performed.

If the provocation is positive, particularly when accompanied by a low tryptase, a non-allergic hypersensitivity can be diagnosed. Other causes that should be considered are the use of disinfectants, medication during procedures and (co-)morbidities. In case of a severe immediate reaction to an ICM based on its osmolarity, it is recommended to switch to an ICM with lower osmolarity. Furthermore, in case of a positive skin test but a negative provocation, no hypersensitivity is diagnosed and the ICM can be used in the future (Figure 2).

In patients with a positive skin test, but without a (typical) hypersensitivity reaction, a provocation with the suspected drug should be performed, particularly because patients can have a positive skin test without a previous reaction to the contrast media.^27,28^ In case of a negative provocation, the patient has no hypersensitivity to the contrast media, while in case of a positive provocation, an allergy is confirmed.

Ideally, no premedication is used during the provocation to enable reliable observation of the type of reaction. Figure 2 represents a proposed flowchart for the assessment of a presumed allergic reaction to contrast media.

This review has several limitations. Studies were either retrospective (10 studies) or prospective and mainly included case series and small cohorts, which can limit the interpretation of the results. Data were summarised and were not pooled in a meta-analysis, because of the heterogeneity in the studies. Furthermore practical guidelines are lacking. None of the studies included details about the provocations such as information on dosage. Moreover, the included studies may have been biased by the use of pre-medication. Four studies reported on the use of premedication (Tables 2–4).^18,21,31,35^ This may decrease the severity of the reaction and therefore influence the results of the provocation test. However, details about the specific premedication were lacking in three of the studies.

Despite these limitations, this review makes a novel contribution to the literature by the proposed flow-chart which could encourage the implementation of provocation as part of the diagnostic work-up in hypersensitivity reactions to contrast media. This proposed flow-chart should be further validated in the future, prior to implementation in practical guidelines.

## Conclusion

In case of IHR and NIHR to ICM, the majority of patients with a positive skin test for the culprit tolerated a challenge with a skin-test-negative alternative ICM. In case of a negative skin test for the culprit ICM, provocations were mostly negative, although the number of positive provocations was higher in the NIHR group. Data on hypersensitivity reactions, skin tests and provocations with gadolinium-based contrast media were limited; however, they exhibited a pattern similar to that observed in ICM. In summary, a thorough medical history is necessary, followed by skin tests. A provocation is recommended for diagnostic work-up, when the diagnosis is uncertain.
